The article "Multiple Statistical Model Ensemble Predictions of Residual Chlorine in Drinking Water: Applications of Various Deep Learning and Machine Learning Algorithms" was published in 2022. Journal: J Environ Public Health.

# Multiple Statistical Model Ensemble Predictions of Residual Chlorine in Drinking Water: Applications of Various Deep Learning and Machine Learning Algorithms

**DOI:** 10.1155/2022/7104752

**Published:** 2022-09-28

**Authors:** Charles Onyutha

**Affiliations:** Department of Civil and Environmental Engineering, Kyambogo University, P.O. Box 1, Kyambogo, Kampala, Uganda

## Abstract

Applicability of statistical models in predicting chlorine decay remains minimally explored. This study predicted residual chlorine using six deep learning and nine machine learning techniques. Suitability of multimodel ensembles (MMEs) including arithmetic mean of all the models (Ens1), average of the best three performing models (Ens2), and weighted mean of outputs from all the 15 models was investigated. A total of nine “goodness-of-fit” measures (such as distance correlation (*r*_d_) and Taylor skill score) were used to rank the models. The two best deep learning methods were the nonlinear autoregressive model with exogenous input (NARX) (*r*_d_ = 0.51) and feedforward backpropagation (FFB) (*r*_d_ = 0.61). The two best machine learning algorithms included random forests (RF) (*r*_d_ = 0.64) and Gaussian process regression (GPR) (*r*_d_ = 0.59). Eventually, Ens2 was obtained using RF, FFB, and GPR. Ens2 performed better than Ens1 and Ens3. The amount of variance explained by individual models and MMEs was over the ranges of 13–66% and 51–74%, respectively. Ens2 explained 74% of the total variance in observed residual chlorine. Remarkably, the appropriateness of the MMEs depends on the approach for combining model outputs, and the number of models considered. This study demonstrated the acceptability of statistical MMEs in predicting chlorine residual concentration in drinking water.

## 1. Introduction

Several drinking water disinfectants exist [1]. Examples of such disinfectants include chlorine dioxide, ozone, ultraviolet light, chloramine, and free chlorine [2]. Free chlorine has several advantages; it is efficacious in disinfection, easy to apply, cheap, and long-lasting, thereby disinfecting water up to the consumer points [1]. Drinking water is recommended to have chlorine residual concentrations in the range 0.2–5 mg/l [3]. Drinking water with concentrations of residual chlorine below 0.2 mg/l tends to be susceptible to regrowth of microbials which infect consumers. On the other hand, overdosage of chlorine can lead to the formation of harmful byproducts such as chloro-organics, haloacetic acids, and trihalomethanes (THM). THM chloroform is known to be carcinogenic to animals [4] and human beings. Other health complications which can result from overdosage of chlorine in drinking water include birth defects and damages to liver and kidney [5]. In places where water distribution networks are ineffectively managed and when treatment plants are outdated or not regularly maintained, careful activities should be designed for monitoring of the system to guard against possible health issues which may arise, for instance, from byproducts of chlorine following overdosage of the chlorine as a disinfectant [6].

The article "Multiple Statistical Model Ensemble Predictions of Residual Chlorine in Drinking Water: Applications of Various Deep Learning and Machine Learning Algorithms" was published in 2022. Journal: J Environ Public Health.

For analysis of how to keep concentrations of residual chlorine in drinking water within the recommended range 0.2–5 mg/l, modelling tends to be conducted. Both physical and statistical models exist for modelling of chlorine decay. Examples of process-based and statistical models include EPANET [7] and artificial neural network, respectively. A recent review showed that 87% and 17% of the studies on modelling chlorine residuals in drinking water applied process-based and statistical models, respectively [2]. Physical models are characterized by scale effects. Furthermore, nontrivial mathematics and several assumptions are required in capturing the behavior of chlorine concentrations under different circumstances of temperature, pH, and other factors. In cases where predictions of residual chlorine concentration (*RCC*) are required given the little available time, data-driven statistical models can be used.

As statistical methods, both machine learning and deep learning techniques can be applied for making predictions of chlorine residual concentrations. Deep learning makes use of deep neural networks. Machine learning comprises the use of computer to train and automate tasks which would turn out to be unbearable or impossible for human beings to perform. Essentially, deep learning is a subset of machine learning. However, both deep learning and machine learning are subsets of artificial intelligence. Worth noting is that the performance of deep learning can differ, to some extent, from that of the machine learning.

Tackling the problem of uncertainties on the modelling outcomes can be undertaken by combining the outputs from various models to obtain one set of modelled results. By combining many realizations from (i) one deterministic model or (ii) various models but of the same structure, we obtain single model ensemble. On the other hand, multimodel ensemble can be obtained from combination of outputs from models of different structural complexity. The application of the concept of multimodel ensemble has been common in hydrological modelling (see, e.g., [8–10]) but not for prediction of chlorine residual in drinking water.

By the time of conducting this research, no any studies could be found in literature to have conducted an in-depth analysis of the prediction of RCC using an array of both machine learning and deep learning techniques while investigating the suitability of multimodel ensemble. Thus, this study is aimed at addressing this knowledge gap in scientific research.

The article "Multiple Statistical Model Ensemble Predictions of Residual Chlorine in Drinking Water: Applications of Various Deep Learning and Machine Learning Algorithms" was published in 2022. Journal: J Environ Public Health.

## 2. Materials and Methods

### 2.1. Methods

#### 2.1.1. Deep Learning

- Nonlinear Autoregressive Model with Exogenous Input (NARX)

To model sequential data, recurrent neural networks (RNNs) can be applied. This is because RNN eliminates the need for having many parameters since it considers each element within the given sequence to be assigned the same weight, something which is not the case for other models such as the deep feedforward model. In an RNN, the exhibition of the temporal dynamic behavior can be linked to the connections among the nodes. The input variable length sequence can be processed based on the internal memory.

NARX [11] is one of the commonly applied RNNs. NARX differs from other networks through its passing of information from one step to another, and it does this by adding loops which feed the preceding inputs and outputs back to the network. NARX also has the typical feature of characterizing lag time of the input and output through the feedback delays [12].

Consider *n*_*x*_ and *n*_*y*_ to denote the number of input and output delays, respectively, such that the actual values of the exogenous inputs include *x*(*t* + 1), *x*(*t*), ⋯, *x*(*t* − *n*_*x*_). Furthermore, let the actual values of the time series be *y*(*t*), *y*(*t* − 1), ⋯, *y*(*t* − *n*_*y*_). If we represent the past estimated or predicted outputs from the NARX model as series $\hat{y}\left(t\right),\hat{y}\left(t-1\right),\cdots ,\hat{y}\left(t-n_{y}\right)$_,_ the typical architectures of NARX [13, 14] can be given by

(1) $$\begin{array}{c} \hat{y}\left(t+1\right)=f\left(y\left(t\right),y\left(t-1\right),\cdots ,y\left(t-n_{y}\right),x\left(t+1\right),x\left(t\right),\cdots ,x\left(t-n_{x}\right)\right), \end{array}$$

(2) $$\begin{array}{c} \hat{y}\left(t+1\right)=f\left(\hat{y}\left(t\right),\hat{y}\left(t-1\right),\cdots ,\hat{y}\left(t-n_{y}\right),x\left(t+1\right),x\left(t\right),\cdots ,x\left(t-n_{x}\right)\right), \end{array}$$

where $\hat{y}\left(t+1\right)$ denotes the predicted output of NARX at the time (*t* + 1), and *f* represents the mapping function. Equation (1) represents the series-parallel (also called open-loop) architecture of NARX. On the other hand, Equation (2) indicates the parallel (also called closed loop) architecture of NARX.

(ii) Long Short-Term Memory (LSTM) Model

LSTM model [15] is another commonly applied RNN. LSTM which is used to effectively capture long-term temporal dependencies has a memory cell as its fundamental structure. The memory cell comprises cell states to remember temporal information. Thus, the memory cell is to remember and propagate unit outputs at various time steps. Flow of information from one time step to another is controlled by the forget gate, input gate, and output gate. Initially, a typical LSTM block comprised the input gate and output gate as well as the cells [15] and the forget gate was not included. Later, the forget gate was introduced into the LSTM architecture by Gers et al. [16], thereby allowing the LSTM to reset its own state.

The article "Multiple Statistical Model Ensemble Predictions of Residual Chlorine in Drinking Water: Applications of Various Deep Learning and Machine Learning Algorithms" was published in 2022. Journal: J Environ Public Health.

Consider that *i*_*t*__,_*o*_*t*__,_ and *f*_*t*_ denote the input gate, output gate, and forget gate, respectively. Furthermore, let *h*_*t*__,_*c*_*t*_^*v*^_,_ and *c*_*t*_ represent the hidden state, candidate vector, and cell state, respectively. Let us also take *b*_*i*__,_*b*_*f*__,_*b*_*o*__,_ and *b*_*c*_ to be the bias for the input gate, forget gate, output gate, and the new cell, respectively. If *x*(*t*) denotes the input vector at time step *t* while *h*_*t*−1_ is the hidden state of the previous time step, the general memory block of the LSTM can be given by *i*_*t*_ = *σ*(*w*_*i*_[*x*(*t*), *h*_*t*−1_] + *b*_*i*_)_,_*f*_*t*_ = *σ*(*w*_*f*_[*h*_*t*−1_, *x*(*t*)] + *b*_*f*_)_,_*o*_*t*_ = *σ*(*w*_*o*_[*h*_*t*−1_, *x*(*t*)] + *b*_*o*_)_,_*c*_*t*_^*v*^ = *σ*(*w*_*c*_[*h*_*t*−1_, *x*(*t*)] + *b*_*c*_)_,_*c*_*t*_ = *f* × *c*_*t*−1_ + *i*_*t*_ × *c*_*t*_^*v*^_,_ and *h*_*t*_ = *o*_*t*_ × tanh(*c*_*t*_) where *σ* and tanh are activation functions.

(iii) Layer Recurrent (LR) Neural Network

LR is another RRN model and was introduced by Xie et al. [17] following the inspiration by the ResNet architecture [18]. LR can adaptively learn contextual information. In the LR architecture, the first step is to compute the local features using the convolutional neural network (CNN) module. In the second step, two 1D spatial RNNs are applied to scan along each of the rows. Thirdly, the two 1D spatial RNNs are applied to scan along each column from two directions [17]. In the LR architecture (see [17] for details), dependencies are captured by the within layer recurrence.

(iv) Feedforward Neural Networks

The main goal of a feedforward neural network (FFN) is to approximate some function. The components of an FFN network include input layer, hidden layer, output layer, and neurons' weights. In FFN, connections among the nodes are not in a circular form. Nodes within the network are used to connect the various units. Information about the network depends on the weight of the connections. The flow of information through the nodes of FFN is in a forward direction. At the neuron output, we have an activation function which serves as the decision-making center.

The article "Multiple Statistical Model Ensemble Predictions of Residual Chlorine in Drinking Water: Applications of Various Deep Learning and Machine Learning Algorithms" was published in 2022. Journal: J Environ Public Health.

After entering the network via the input point, the data passes through each and every layer of the network before obtaining the outputs. At first, the set of inputs are multiplied by their weights after entering through the input layer. The second step consists of summing up the weighted inputs such that we can have the output as 1 (if the sum of the value exceeds a specified threshold) or -1 (when the value is exceeded by the limit). The third step comprises classification and here, concepts of machine learning can be applied for the classification. In the fourth step, outputs can be compared with the predicted values. At this point, the training procedure ensures weights are optimized to enhance accuracy. The last step consists of backpropagation in which the weights are updated especially in a multilayered networks and hence, the name feedforward backpropagation (FFB) neural network. Instead of backpropagation, we can have a tap delay line associated with each input and weights and in this line, we talk about the feedforward distributed time delay (FFDT) neural network.

(v) Adaptive-Network-Based Fuzzy Inference System (ANFIS)

ANFIS is some kind of artificial neural network [19]. It integrates neural networks and fuzzy logic. The learning capability of ANFIS in approximating nonlinear functions can be linked to the set of fuzzy if–then rules.

ANFIS applies a hybrid learning rule to combine the least squares method and backpropagation gradient descent [19] in identifying an array of parameters for generating the previously obtained input-output pairs. The neural fuzzy control system used for the ANFIS was based on the Takagi-Sugeno-Kang fuzzy rules in the form

(3) $$\begin{array}{c} R_{1}:\text{If }x_{1}\text{ is }C_{1}^{1}\text{ and }x_{2}\text{ is }C_{1}^{2},\text{then }y=f_{1}=c_{0}^{1}+c_{1}^{1}x_{1}+c_{2}^{1}x_{2},\\ R_{2}:\text{If }x_{1}\text{ is }C_{1}^{2}\text{ and }x_{2}\text{ is }C_{1}^{2},\text{then }y=f_{2}=c_{0}^{2}+c_{1}^{2}x_{1}+c_{2}^{2}x_{2}, \end{array}$$

and for the two inputs, *x*_1_ and *x*_2__,_ the inferred output *y*^#^ = (*γ*_1_*f*_1_ + *γ*_2_*f*_2_)/(*γ*_1_ + *γ*_2_) where *γ*_*j*_ denotes the firing strengths of *R*_*j*_(*j* = 1, 2) and can be computed using *γ*_*j*_ = *γ*_*C*_1_^*j*^_(*x*_1_) × *γ*_*C*_2_^*j*^_(*x*_2_).

We can consider ANFIS to have 5 layers. The first layer is actually an adaptive node comprising a node function. In the second layer, all the incoming signals are multiplied to obtain an output. In layer 3, the ratio of the *i*^th^ rule's firing strength to the sum of all the various rules' firing strength is computed and in this layer we consider each node to be fixed. In layer 4, each node is taken to be an adaptive node and comprises a node function. It is in layer 5 that we compute the overall output by adding all the incoming signals and to do so, each node is considered fixed.

The article "Multiple Statistical Model Ensemble Predictions of Residual Chlorine in Drinking Water: Applications of Various Deep Learning and Machine Learning Algorithms" was published in 2022. Journal: J Environ Public Health.

#### 2.1.2. Machine Learning

- Randomforest (RF) Regression

RF developed by Breiman [20] comprises a methodology in which results from decision trees are averaged to obtain a better outcome. Here, the decision trees can be thought of in terms of a number of weak heterogeneous individual learners who are trained. Given a complex problem, we believe that these learners (as a group) can make better decision than (expert) individuals. Thus, the decision tree represents an outcome obtained by combining the results of the learners in a manner, for instance, through a voting scheme to ensure the overall result typifies an enhanced yield.

Recursive partitioning is applied to establish a regression tree. Bagging (which is the process of creating training data through random sampling with replacement) is used to minimize the diversity of trees. The out-of-bag (or the subset of trees which are not selected as training data in the bagging process) are used for checking model's performance.

Consider *N* to be the number of samples while *M* denotes the attributes or the number of input features. Furthermore, let *ψ* be the total number of trees to be grown to become a forest. Bootstrap sampling is performed for each tree in a forest to come up with *N* samples. In the sampling procedure, samples are selected randomly and this is done with replacement. To grow a new decision tree for every training set, the CART method of Breiman et al. [21] can be used. It is from the node that a new split can occur. To do so, we consider only *q* number of features such that *q* is less than *M*, for instance, $q=\sqrt{M}.$ We repeat this process several times until a total of *ψ* trees are obtained to comprise a random forest. The last step is the decision which entails averaging the tree predictions.

(ii) Support Vector Machine (SVM)

The idea of the Support Vector Machine (also known as the classification and regression procedure) is that it should map the input vectors into high dimensional feature space [22] and this is to simplify classification problem in the feature space. In a high dimensional feature space mapped from the input data using the device called kernel mapping, the problem can become linearly separable [23]. SVM has commendable capacity in establishing unknown relationships which may exist between a set of various input variables and the system output. The key aspect of SVM which makes it so advantageous is the use of a kernel trick for establishing knowledge about a given problem in a manner that can allow both model residuals (or prediction errors) and the model complexity to be minimized in a simultaneous way.

The article "Multiple Statistical Model Ensemble Predictions of Residual Chlorine in Drinking Water: Applications of Various Deep Learning and Machine Learning Algorithms" was published in 2022. Journal: J Environ Public Health.

Let us assume that we have a training dataset (**x**, *y*) such that **x** ∈ *ℜ*^*n*^ and *y* ∈ *ℜ* where *ℜ* denotes the input space with **x** = {**x**_1_, **x**_2_, ⋯} as the input vector while *y* is the system output [24]. If **v** represents the matrix of regression weights while *b* is the bias term (which denotes the threshold in the support vector machines), to obtain a function *f* with small risk using an independent uniformly distributed dataset (**x**_1_, *y*_1_),...., (**x**_*n*_, *y*_*n*_), we can, by some nonlinear mapping *Φ*, *map ***x** into the feature space [25] with the nonlinear estimate function given by *y* = *f*(**x**, **v**) = **v**^T^*Φ*(**x**) + *b*. Following Vapnik [22] and Cortes and Vapnik [26], regularized risk functional for obtaining small risk can be given in terms of the penalty parameter (*D*), number of support vectors (*n*^∗^), small positive number (*G*), and support vectors obtained from training data (**x**_*i*_) such that

(4) $$\begin{array}{c} \frac{1}{2}{\left\|v\right\|}^{2}+\frac{D}{n^{*}}\overset{n^{*}}{\underset{i=1}{\sum }}{\left|y_{i}-f\left(x_{i},v\right)\right|}_{G}. \end{array}$$

If (*β*_*i*_^#^, *β*_*n*_) denotes coefficients which can be determined by training, while *K*(**x**_*i*_, **x**_*j*_) is the support vector kernel, we can form a kernel to satisfy the Mercer's condition or a dot-product kernel by *K*(**x**, **x**′) = *K*(〈**x**.**x**′〉) [27]. Equation (4) leads us to dual optimization problem in which we have to

(5) $$\begin{array}{c} \text{Maximize }W\left(\beta^{\#}\right)=-G\times \overset{n^{*}}{\underset{i=1}{\sum }}\left(\beta_{i}^{\#}+\beta_{i}\right)+\overset{n^{*}}{\underset{i=1}{\sum }}\left(\beta_{i}^{\#}-\beta_{i}\right)y_{i}-\frac{1}{2}\overset{n^{*}}{\underset{i=1}{\sum }}\overset{n^{*}}{\underset{j=1}{\sum }}\left(\beta_{i}^{\#}-\beta_{i}\right)\left(\beta_{j}^{\#}-\beta_{j}\right)K\left(x_{i}.x_{j}\right).\\ \begin{array}{c} \text{subject to}\\ \overset{n^{*}}{\underset{i=1}{\sum }}\left(\beta_{i}^{\#}-\beta_{i}\right)=0\;\beta_{i}^{\#}\in \left[0,D\right] \end{array} \end{array}$$

Finally, the decision function can be given by *f*(**x**) = ∑_*i*=1_^*n*^∗^^(*β*_*i*_^#^ − *β*_*i*_)*K*(**x**, **x**′) + *b*_,_ such that the *K*(**x**, **x**′)_,_ as normally taken to be the Gaussian kernel, is computed using

(6) $$\begin{array}{c} K\left(x,x^{\prime }\right)=\exp\left(-\frac{{\left\|x-x^{\prime }\right\|}^{2}}{2\sigma^{2}}\right). \end{array}$$

(iii) Generalized Linear Models (GLMs)

GLMs consist of a modelling framework which lead to a family of models. Each of the family members makes use of a particular link function and specific distribution. A link function is used to mathematically establish the linearity. The outcome variable can be fitted using a particular distribution. What is important here is the selection of the shape which can match the given randomness and in this way, we can eliminate the tough assumption of a constant variance. There are several distributions which tend to be used. For instance, this study employed GLMs based on beta distribution (GLMB), normal distribution (GLMN), poisson distribution (GLMP), gamma distribution (GLMG), and inverse Gaussian distribution (GLMI).

(iv) Discriminant Analysis Model (DAM)

Discriminant analysis is a natural technique to make forecast especially when the predictand comprises a finite set of discrete groups given that vectors of predictors are known. The discriminant analysis as a classification technique relies on the assumption that different classes can be generated based on different Gaussian distributions. Discriminant analysis can be applied to characterize differences between groups and use the characteristics for classification of a new member to be added to the groups, and this is based on the observations obtained from the member. In discriminant analysis, a member is characterized using a vector of variables which comprise a multivariate density function. The multidimensional characteristics of the density function of the population's variable are mapped onto a one dimensional measure using a discriminant function.

The article "Multiple Statistical Model Ensemble Predictions of Residual Chlorine in Drinking Water: Applications of Various Deep Learning and Machine Learning Algorithms" was published in 2022. Journal: J Environ Public Health.

In a DAM, the predictor **x** is assumed to have a Gaussian mixture distribution. For DAM, two options exist including linear discriminant analysis and quadratic discriminant analysis. In the former case, we assume that only the means vary while each class has the same covariance matrix. In the latter case, both covariance and the mean of every class vary. In training a classifier, parameters of a Gaussian distribution for every class are estimated using a suitable fitting function. For predicting the classes of new data, the trained classifier determines the class which has the smallest misclassification cost.

(v) Gaussian Process Regression (GPR)

GPR model is a nonparametric kernel-based probabilistic model. Let *n* be the sample size. If we have a training dataset {(*x*_*i*_, *y*_*i*_); *i* = 1, 2, ⋯, *n*} such that *t*, *x*_*i*_ ∈ *ℜ*^*n*^, and *y*_*i*_ ∈ *ℜ* all drawn from an unknown distribution, we can use GPR to predict the system output *y* given the new input vector **x**. We can make use of a linear regression of the form *y* = *x*^*T*^*α* + *ε* such that *ε* ~ *N*(0, *σ*^2^). The data can be used to estimate the coefficient *α* and the error covariance *σ*^2^. To explain the response of the system, GRP introduces (i) explicit basis function *h* to project the predictors or inputs *x*_*i*_ into p-dimensional feature space and (ii) the set of latent variables *f*(*x*_*i*_); 1 ≤ *i* ≤ *n* from a Gaussian process for capturing the smoothness of the system response.

The article "Multiple Statistical Model Ensemble Predictions of Residual Chlorine in Drinking Water: Applications of Various Deep Learning and Machine Learning Algorithms" was published in 2022. Journal: J Environ Public Health.

A GPR model may be represented as *h*(*x*)^*T*^*α* + *f*(*x*), such that *f*(*x*) ~ Gaussian process with mean = 0 and covariance = *K*(*x*, *x*′). The system response *y* can be modelled using

(7) $$\begin{array}{c} P\left(y_{i}\left|f\left(x_{i}\right),x_{i}\right.\right)\sim N\left(y_{i}\left|h{\left(x_{i}\right)}^{T}\right.\alpha +f\left(x_{i}\right),\sigma^{2}\right). \end{array}$$

#### 2.1.3. Water Quality Data

To evaluate the performance of the various models, water quality datasets based on samples taken from the Lirima Gravity Flow Scheme (LGFS) in Uganda, East Africa, were used. The LGFS is owned and operated by the National Water and Sewerage Corporation (NWSC) as a utility parastatal under sole ownership of the Government of Uganda. NWSC is known for its commitment for the provision of clean and safe water in the various towns, cities, and urban centers across Uganda. Sampling and testing water from the LGFS (which is about 90 km in length) for this research followed a formal permission granted by the Research and Development Department from the Head Office of the NWSC in Kampala.

Several points were selected within the LGFS for water sampling. At each location or point, water was sampled several times (both in the morning and afternoon) within each day. From each water sample, several water quality parameters were tested and recorded including water temperature (°C), pH, electrical conductivity (*μ*S), and RCC (mg/l). These factors were reported to influence decay of chlorine (see, e.g., [2, 28–31]), and they were deemed to be possible predictors of RCC.

It is important to recall that chlorine decay depends on time and this follows the kinetic of chlorine reaction with water as governed by the first order equation *C*_res_(*t*) = *C*_ini_ × exp(−*K*_*b*_ × *t*) where *C*_res_(*t*) is the RCC (mg/l) at time *t*, *C*_ini_ denotes the chlorine concentration (mg/l) at time *t* = 0_,_ and *K*_*b*_ refers to the chlorine bulk reaction constant (measured per hour). Thus, the time *t* at which the water was sampled was also recorded. Eventually, water temperature (°C), pH, electrical conductivity (*μ*S), and the sampling time were considered as predictors (*X*_1__,_*X*_2__,_*X*_3__,_ and *X*_4__,_ respectively) of the RCC. To do so, *X*_4_ was converted from the format of an hour (e.g., 13 : 00 hours) to become a number (i.e., 0.54) and this was done using an in-built function (or option for number formatting) in the Ms Excel.

The article "Multiple Statistical Model Ensemble Predictions of Residual Chlorine in Drinking Water: Applications of Various Deep Learning and Machine Learning Algorithms" was published in 2022. Journal: J Environ Public Health.

#### 2.1.4. Training and Testing of the Various Models

Performance of each of the various deep learning and machine learning algorithms was assessed using several “goodness-of-fit” metrics including the coefficient of determination (*R*^2^ or R-squared), revised R-squared (RRS, [32]), Nash Sutcliffe efficiency [33], hydrological model skill score or Onyutha efficiency (OE, [32]), root mean square error (RMSE), percentage bias (PBIAS), symmetric mean absolute percentage error (SMAPE), index of agreement (IOA, [34]), Taylor skill score (TSS, [35]), and distance correlation (*r*_*d*_, [36]). Based on the observed (*x*) and modelled (*y*) RCC, consider some of the relevant terms of these “goodness-of-fit” metrics to be sample size (*n*), mean of *x*$\left(\bar{x}\right)$, mean of *y*$\left(\bar{y}\right)$, variance of *x*(s_x_^2^), variance of *y*(s_y_^2^), standard deviation of *x*(s_*x*_), standard deviation of *y*(s_*y*_), normalized *s*_*y*_$\left({\hat{s}}_{y}\right)$, distance covariance of *x*(d_*xx*_), distance covariance of *y*(d_*yy*_), distance covariance of *x* and *y*(d_*xy*_), maximum correlation attainable (*r*_*m*_) (in this study *r*_*m*_ was set to 0.99), and variance of *y* constrained to $\bar{x}$ as the comparison baseline (*s*_*yc*_^2^) such that ${\text{s}}_{yc}^{2}={\left(n-1\right)}^{-1}\times \sum_{i=1}^{n}{\left(y-\bar{x}\right)}^{2}$. The various measures to assess model performance were computed using the following

(8) $$\begin{array}{c} R^{2}=\frac{\sum_{i=1}^{n}\left(x_{i}-\bar{x}\right)\left(y_{i}-\bar{y}\right)}{\sqrt{\sum_{i=1}^{n}{\left(x_{i}-\bar{x}\right)}^{2}\sum_{i=1}^{n}{\left(y_{i}-\bar{y}\right)}^{2}}}, \end{array}$$

(9) $$\begin{array}{c} \text{RRS}=\left|r\right|\times \frac{\min\left({\text{s}}_{\text{x}},{\text{s}}_{\text{y}}\right)}{\max\left({\text{s}}_{\text{x}},{\text{s}}_{\text{y}}\right)}\times \frac{\min\left({\text{s}}_{\text{x}}^{2},{\text{s}}_{yc}^{2}\right)}{\max\left({\text{s}}_{\text{x}}^{2},{\text{s}}_{yc}^{2}\right)}, \end{array}$$

(10) $$\begin{array}{c} \text{NSE}=1-\frac{\sum_{i=1}^{n}{\left(x_{i}-y_{i}\right)}^{2}}{\sum_{i=1}^{n}{\left(x_{i}-\bar{x}\right)}^{2}}, \end{array}$$

(11) $$\begin{array}{c} r_{d}=\frac{{\text{d}}_{\text{xy}}}{\sqrt{{\text{d}}_{\text{xx}}\times {\text{d}}_{\text{yy}}}}, \end{array}$$

(12) $$\begin{array}{c} \text{OE}=r_{d}\times \frac{\min\left({\text{d}}_{\text{XX}},{\text{d}}_{\text{YY}}\right)}{\max\left({\text{d}}_{\text{XX}},{\text{d}}_{\text{YY}}\right)}\times \frac{\min\left({\text{s}}_{\text{x}}^{2},{\text{s}}_{yc}^{2}\right)}{\max\left({\text{s}}_{\text{x}}^{2},{\text{s}}_{yc}^{2}\right)}, \end{array}$$

(13) $$\begin{array}{c} \text{IOA}=1-\frac{\sum_{i=1}^{n}{\left(x_{i}-y_{i}\right)}^{2}}{\sum_{i=1}^{n}{\left(\left|\left(x_{i}-\bar{x}\right)\right|+\left|\left(y_{i}-\bar{y}\right)\right|\right)}^{2}}, \end{array}$$

(14) $$\begin{array}{c} \text{TSS}=\frac{4\left(1+{\left(n\times s_{x}s_{y}\right)}^{-1}\sum_{i=1}^{n}\left(x_{i}-\bar{x}\right)\left(y_{i}-\bar{y}\right)\right)}{{\left({\overset{\wedge }{s}}_{y}+{\left({\overset{\wedge }{s}}_{y}\right)}^{-1}\right)}^{2}\left(1+r_{m}\right)}, \end{array}$$

(15) $$\begin{array}{c} \text{RMSE}=\sqrt{\frac{1}{n}\overset{n}{\underset{i=1}{\sum }}{\left(x_{i}-y_{i}\right)}^{2}}, \end{array}$$

(16) $$\begin{array}{c} \text{SMAPE}=\frac{100}{n}\times \overset{n}{\underset{i=1}{\sum }}\frac{\left|x_{i}-y_{i}\right|}{\left|x_{i}\right|+\left|y_{i}\right|}, \end{array}$$

(17) $$\begin{array}{c} \text{PBIAS}=\frac{100\times \sum_{i=1}^{n}\left(x_{i}-y_{i}\right)}{\sum_{i=1}^{n}x_{i}}. \end{array}$$

In Equations (9) and (12), min () denotes whichever is smaller of the two values. Each of the modelling datasets was divided into training (70%) and testing (30%) subseries. Model performance evaluation was conducted using (i) training data, (ii) testing data, and (iii) entire data (when both training and testing series were combined). Each of the “goodness-of-fit” metrics (Equations (8)–(17)) was applied to evaluate the outputs of the various deep learning and machine learning models. To download the MATLAB codes for computing RRS (Equation 9) and OE (Equation 12), the reader is referred to https://doi.org/10.5281/zenodo.6570904 and the access is unrestricted.

The article "Multiple Statistical Model Ensemble Predictions of Residual Chlorine in Drinking Water: Applications of Various Deep Learning and Machine Learning Algorithms" was published in 2022. Journal: J Environ Public Health.

The next step comprised ranking the models to indicate which one was the best or the worst in terms of performance to reproduce the available observations. Based on the values of a particular “goodness-of-fit” metric, models were ranked. Each of the metrics in Equations (8), (9), and (11)–(14) varies from zero to one. A value of zero shows the worst model performance. For an ideal model (or one with the best performance), each of these metrics (Equations (8), (9), and (11)–(14)) gives a value of one. The best and worst model performance is shown by NSE (Equation (10)) values of one and negative infinity, respectively. However, for RMSE, SMAPE, and PBIAS (Equations (15)–(17)), the best model performance can be obtained when the value of the “goodness-of-fit” metric is zero. When there are many models, the one with the largest value of RMSE indicates the worst model fit. The same is true when we consider each of the metrics SMAPE and PBIAS (Equations (16) and (17)). Therefore, for each of the metrics in Equations (8)–(14), ranks of 1, 2,….., *w* were given to the model with the highest, second highest, ...., lowest value, respectively, of the “goodness-of-fit” metric under consideration. However, for statistical metrics in Equations (15)–(17), ranks of 1, 2,….., *w* were given to the model with lowest, second lowest,….., highest value, respectively, of a particular “goodness-of-fit” metric.

Let *η*to denote the number of “goodness-of-fit” metrics (and this was 10 in this study). Ranks of each of the fifteen models based on assessments from the various “goodness-of-fit” metrics were summed up. This resulted into a total of *w* (or 15) values which were expected to vary between (*η* − 1) to ((*η* × *w*) + 1). Finally, the sums of the ranks were sorted in ascending order. The model with the smallest sum, second smallest sum, ...., and the largest sum was given performance index 1, 2,….., *w*, (as the best, second best,….., worst model), respectively.

#### 2.1.5. Developing Ensemble Predictions

There are various ways of obtaining model ensembles such as simple model average, weighted average method, multiple super model ensemble, and constrained multiple linear regression. For brevity, this study examined the suitability of three model ensembles including the arithmetic model average of all the modelled results (Ens1), arithmetic mean of results from the best three models (Ens2), and weighted mean of outputs from all the models (Ens3). Consider *y*_*i*_^(*j*)^ as the *j*^*th*^ output of the *i*^*th*^ model, Ens1 was computed using

(18) $$\begin{array}{c} \text{Ens}1_{j}=\frac{1}{w}\overset{w}{\underset{i=1}{\sum }}y_{i}^{\left(j\right)}\;\text{for}\;1\leq j\leq n. \end{array}$$

Ens2 was also computed using Equation (18) with *w* set to 3 (i.e., the first, second, and third best performing models). Let *r*_*d*(*i*)_ be the distance correlation between the observed data and outputs of the *i*^*th*^ model while *p* is the absolute value of an arbitrary power (and *p* was set to 15 in this study). It is worth noting that *p* depends on the magnitudes of the values in the series. Ens3 was computed using

(19) $$\begin{array}{c} \text{Ens}3_{j}=\frac{\sum_{i=1}^{w}\left(y_{i}^{\left(j\right)}\times {\left(r_{d\left(i\right)}\right)}^{p}\right)}{\sum_{i=1}^{w}{\left(r_{d\left(i\right)}\right)}^{p}}\;\text{for}\;1\leq j\leq n. \end{array}$$

## 3. Results

Figure 1 shows performance of the various statistical models in reproducing observed RCC. Notably, the performance depends on the selected “goodness-of-fit” metric (Figure 1). This is because of the differences among the “goodness-of-fit” metrics. For instance, some metrics like NSE, IOA, and RMSE are based on squared model residuals while RSS and OE consider combined measures of variability, bias, and correlation. Furthermore, the various objective functions differ in terms of their ranges over which their values occur. For instance, NSE ranges from negative infinity to one while R^2^, RRS, OE, TSS, IOA, and *r*_*d*_ occur over the range 0–1. Values of RMSE range from zero to positive infinity. However, the RMSE values were all small in magnitude and one may associate these values to a possible excellent performance of the models. Nevertheless, it should be noted that the small values of RMSE were due to the small values of the RCC. For instance, the observed RCCs ranged from 0.01 to 0.48 mg/l with an average of 0.14 mg/l. For all the models, some metrics especially TSS and IOA exhibited values which were close to one (indicating best model performance). The sensitivity of IOA in yielding values close to one even for models which is characterized by poor fit was shown by Krause et al. [37]. The tendency of TSS to yield values close to 1 for models which are not perfect was also recently obtained by Onyutha [32].

The article "Multiple Statistical Model Ensemble Predictions of Residual Chlorine in Drinking Water: Applications of Various Deep Learning and Machine Learning Algorithms" was published in 2022. Journal: J Environ Public Health.

Considering the average of each “goodness-of-fit” metric, the deep leaning methods (NARX, FFB, FFDT, LR, ANFIS, and LSTM) were generally better than the machine learning techniques (RF, SVM, DAM, GLMB, GLMN, GLMP, GLMG, GLMI, and GPR). The best two performing machine learning methods included RF and GPR. On the other hand, FFB and NARX were the two best deep learning methods. In most cases, model results of training were slightly better than those for testing. Furthermore, models evaluated using the entire data (both calibration and testing subseries) were found to perform better than when testing subseries were used.

Figure 2 shows results of error analysis. For each model, the errors were mainly concentrated around zero. Values ranging from -0.1 to 0 were greater in number than those over the range 0-0.1 (Figures 2(a) and 2(b)). The median lines of the boxplots for the various models are notably around or close to zero. These impressions can suggest that the models exhibited very high performance. However, by realizing that the actual observed (target) data against which each model was being calibrated ranged from 0.01 to 0.48 mg/l, it means that the impressive performance was due to the order of magnitude of the values being considered (Figure 2(b)). The difference between two small values is even smaller. Nevertheless, it is noticeable that the whiskers of the boxplots of the models go beyond the absolute value of 0.2 mg/l. This suggest that large observed values were mainly either overestimated or underestimated. Based on the results for graphical error analysis, the best performing models were FFB, RF, and GPR (Figure 2(b)). This, however, could not be conclusive without further analysis of the model performances as done next.

The article "Multiple Statistical Model Ensemble Predictions of Residual Chlorine in Drinking Water: Applications of Various Deep Learning and Machine Learning Algorithms" was published in 2022. Journal: J Environ Public Health.

Figure 3 shows comparison of observations with model outputs. Each of the charts (Figures 3(a)–3(o)) contains the 1 : 1 or *y* = *x* diagonal line through the scatter points. For an effective model, all the scatter points would fall along the bisector (or diagonal line). For deep learning methods (Figures 3(a)–3(f)) and three of the machine learning techniques including RF, SVM, and GPR (Figures 3(g)–3(h), (o)), the scatter points especially for RCC values lower than 0.3 mg/l were distributed above and below the bisector. The scatter points from DAM were more widely distributed than those of other models. For the remaining machine learning techniques (Figures 3(j)–3(n)), the scatter points tended to be distributed horizontally between the lines *y* = 0 and *y* = 0.2 mg/l. The scatter points especially, for RCC values greater than 0.3 mg/l, were characterized by large spread around the bisector. One cause of this would be heteroscedascticity or the existence of increasing differences among observations. However, a close look at the scatter points shows that the large values were instead systematically underestimated. Thus, the large spread of the large values were indicative of the difficulty of the models to reproduce observations especially as the RCC increased in magnitude.

Figure 4 shows the heat map for the model performance evaluation. On average, the deep learning methods generally performed better that the machine learning techniques. For instance, the ranks obtained for the GLMs based on beta (GLMB), normal (GLMN), poisson (GLMP), gamma (GLMG), and inverse Gaussian (GLMI) distributions were large. This is consistent with the poor performance of these models as already demonstrated in Figures 1–3.

Evidently, there was no any model which scored the same rank considering all the metrics used to measure model quality. This indicates that the judgement of a model depends on the selected “goodness-of-fit” metric.

Figure 5 shows the overall summary of the model performance. The two best performing machine learning methods included RF and GPR (Figure 4(a)). On the other hand, NARX and FFB yielded the best performance compared with the other deep learning models (Figure 4(b)). When all the models were considered, the ranking process showed that the first, second, third, and fourth best models were RF, FFB, GPR, and NARX, respectively (Figure 4(c)).

The article "Multiple Statistical Model Ensemble Predictions of Residual Chlorine in Drinking Water: Applications of Various Deep Learning and Machine Learning Algorithms" was published in 2022. Journal: J Environ Public Health.

Generally, the best performing GLM was that based on the normal distribution. Nevertheless, the GLMs did not generally perform well compared with other models. In summary, DAM, GLMI, GLMP, and GLMP were the four worst performing models, and they were all based on the machine learning techniques.

Figure 6 shows comparison of ensembles with observed RCC. Observed values from 0.3 mg/l and above were mainly underestimated by each of the model ensembles. This showed lack of capacity of the models to capture large RCCs. Results of the statistical measures of the mismatches between observed and ensemble RCC can be seen in Table 1. As already shown in Figure 4, RF was the best model. However, each set of the model ensembles performed better than RF (Table 1). This demonstrated the need to prefer model ensembles to results of individual models. Ens2 (or arithmetic mean of results from the top or best 20% of the 15 models) exhibited the best performance. This was followed by Ens2 (or weighted mean from all the 15 models).

## 4. Discussion

Application of statistical models is on the increase in a number of areas such as prediction of precipitation ([12, 38–42], river flow ([43–47]), and temperature ([48, 49], and [50]). Some recent studies on modelling water quality using statistical methods include Wadkar and Kote [51], Li et al. [52], García-Ávila et al. [29], and De Santi et al. [53]). For predicting RCC in drinking water, most of the studies (about 90%) available in literature as shown by Onyutha and Kwio-Tamale [2] applied artificial neural networks. Examples of such studies include Wadkar and Kote [51], and García-Ávila et al. [29]. As demonstrated in this study, both machine learning and deep learning methods (which are actually subsets of artificial intelligence) can be applied for making predictions of RCC. Machine learning techniques can fall under four main categories including (i) semisupervised learning, (ii) unsupervised learning, (iii) supervised learning, and (iv) reinforcement learning. The key issues with the machine learning is that it requires selection of features which must carefully be done before the process of training can be performed. This follows from the selectivity invariance issues to which machine learning techniques are susceptible. On the other hand, deep learning eliminates the requirement of feature selection by making use of various abstraction layers to automatically learn the details of the data through application of nonlinear techniques to solve complex problems.

A reliable insight on the uncertainty on modelling results due to the choice of a particular model can be obtained when many models are applied. It is known that each of the various models could be characterized by varying degree of structural complexity. Thus, combining outputs from various models to obtain one set (or an ensemble) of modelled results is important to take into account the uncertainties due to the differences among models. The concept of multimodel ensemble has not been applied in predictions of RCC in drinking water. However, as demonstrated in this study, a multimodel ensemble can perform better than outputs from individual models thereby boosting the credibility and confidence in the predictions of RCC in drinking water.

The article "Multiple Statistical Model Ensemble Predictions of Residual Chlorine in Drinking Water: Applications of Various Deep Learning and Machine Learning Algorithms" was published in 2022. Journal: J Environ Public Health.

While modelling chlorine residuals, most modelers tend to make use of the R^2^ or R-squared [2]. The use of R^2^ is premised on the assumption that the relationship between the predictor and predictand is linear. Thus, the value of R^2^ becomes wrong when we have nonlinear relationships. Other commonly used “goodness-of-fit” metrics include RMSE and mean squared error (MSE). By squaring the model residuals, large weights are assigned to big values and this makes RMSE and MSE sensitive to outliers. As shown in this study, the choice of a particular “goodness-of-fit” metric influences the selection of the best performing model. Thus, it is important to conduct comparative analysis of models while taking into consideration the influence of the choice of a particular objective function or “goodness-of-fit” metric in judging the quality of each model. Several objective functions can be considered including, among others, RRS [32], NSE [33], OE [32], PBIAS, SMAPE, IOA [34], TSS [35], and *r*_*d*_ [36]. Results of a careful intercomparison of models conducted to select the best performing models can crucially influence the suitability of a multimodel ensemble.

## 5. Conclusions

Following the limited exploration of the applicability of the statistical models for modelling chlorine decay, this study investigated the performance of deep learning and machine learning methods in predicting chlorine residuals in drinking water. Suitability of arithmetic mean of all the models (Ens1), average of the best three performing models (Ens2), and weighted mean of outputs from all the 15 models applied in this study was investigated. Generally, on average, results of deep learning methods were better than those of the machine learning techniques. Considering only the deep learning algorithms, the first and second best methods were NARX and FFB, respectively. If we consider only the machine learning algorithms, the first and second best methods included RF and GPR, respectively. The worst deep learning method and machine learning techniques included the LR neural network and DAM, respectively. By combining all the machine learning and deep learning algorithms, the first, second, and third best methods included RF, FFB, and GPR, respectively.

The article "Multiple Statistical Model Ensemble Predictions of Residual Chlorine in Drinking Water: Applications of Various Deep Learning and Machine Learning Algorithms" was published in 2022. Journal: J Environ Public Health.

The total variance explained by the individual models ranged from 13% to 66%. However, multimodel ensembles explained total variance in the range 51-74%. Ens2 explained 74% of the total variance in observed residual chlorine. Thus, the performance of Ens2 was better than that for each of the individual models.

This study corroborated the acceptability of multimodel ensemble prediction of chlorine residual concentrations in drinking water. It is important that intercomparison of models should carefully be conducted to select the best model which can be applied. Comparison of the models should be based on a number of model efficiency criteria. This is because, the use of a particular “goodness-of-fit” metric influences the judgement of model quality.

## Figures and Tables

**Figure 1:** Values of “goodness-of-fit” metrics for (a) training, (b) validation, and (c) entire data.

**Figure 2:** Error analysis based on (a) histogram and (b) boxplots.

**Figure 3:** Observed versus modelled RCC based on (a)–(f) deep learning and (g)–(o) machine learning methods.

**Figure 4:** Performance of models considering (a) machine learning, (b) deep learning, and (c) combination of both machine learning and deep learning methods.

**Figure 5:** Overall performance of models.

**Figure 6:** Observed versus modelled RCC for ensemble model.

**Table 1:** Performance of the model ensembles.

Metric	Ens1	Ens2	Ens3
R^2^	0.507	0.736	0.731
Rr	0.170	0.360	0.356
E	0.081	0.223	0.218
RMSE	0.073	0.054	0.055
PBIAS	13.237	10.280	10.416
NSE	0.443	0.691	0.685
SMAPE	20.834	16.286	16.402
TSS1	0.658	0.844	0.841
IOA1	0.763	0.893	0.891
*r*_d_	0.509	0.708	0.703

## Data Availability

Data used in this study can be obtained upon request from the corresponding author.

## Abbreviations

ANFIS: Adaptive-network-based fuzzy inference system
DAM: Discriminant analysis model
FFN: Feedforward neural network
GLM: Generalized linear model
GLMB: GLM based on beta distribution
GLMG: GLM based on gamma distribution
GLMI: GLM based on inverse Gaussian distribution
GLMN: GLM based on normal distribution
GLMP: GLM based on poisson distribution
GPR: Gaussian process regression
IOA: Index of agreement
LGFS: Lirima gravity flow scheme
LSTM: Long short-term memory
NARX: Nonlinear autoregressive model with exogenous input
NSE: Nash-Sutcliffe efficiency
NWSC: National water and sewerage corporation
OE: Onyutha efficiency
PBIAS: Percentage bias
RCC: Residual chlorine concentration
RF: Randomforest
RMSE: Root mean square error
RNNs: Recurrent neural networks
RRS: Revised R-squared
SMAPE: Symmetric mean absolute percentage error
SVM: Support vector machine
TSS: Taylor skill score.
